# Heterogeneous Multi UAV Mission Planning Based on Ant Colony Algorithm Powered BP Neural Network

**DOI:** 10.1155/2021/4369201

**Published:** 2021-12-02

**Authors:** Wei Tan, Yongjiang Hu, Yuefei Zhao, Wenguang Li, Yongke Li, Xiaomeng Zhang

**Affiliations:** Department of UAV Engineering, Shijiazhuang Campus, Army Engineering University, Hebei, Shijiazhuang 050051, China

## Abstract

With the development of modern science and technology, the field of UAV has also entered the era of high-tech exploration. Among them, the task planning, allocation, path exploration, and algorithm optimization of heterogeneous multi UAV technology are our main concerns. Based on the above situation, this paper proposes a heterogeneous multi UAV task planning technology based on ant colony algorithm powered BP neural network. The planning, research, and design are mainly carried out according to the actual situation of the UAV flight test, and the mathematical programming model is established according to the UAV load degree and maximum flight distance as constraints. This paper focuses on the contribution of the ant colony optimization algorithm to benefit maximization and task minimization. The experimental results show that the BP neural network optimized by the ant colony algorithm can improve the number of iterations and training time. Compared with some comparative algorithms, its performance is better.

## 1. Introduction

With the rapid development and in-depth research of science and technology and neural network technology, the combination of UAV and the above technologies has also become one of the important contents of people's attention. Since the invention of the first UAV in 1971, UAVs have been used in all walks of life, such as military defense, military reconnaissance, greenhouse gas detection, agricultural planting, and material transportation in natural disasters [1]. The reason why UAV technology is widely used as the support of field development mainly stems from its low cost, high safety, durability, and self-operability [2, 3]. However, in the process of UAV use, it will face many problems, the most critical of which is the task execution. We will face the problems that the UAV cannot get our feedback instructions in time and effectively and cannot optimize and allocate the task path, resulting in too slow operation efficiency. Therefore, how to effectively plan the mission path, allocate flight time, obtain the best flight path, and automate the mission planning in the process of mission execution is the key development and optimization of UAV technology [4].

At present, in the use of UAV, when the real environment and main tasks are complex, it is difficult to complete the established tasks efficiently and effectively by only one UAV [5, 6]. Therefore, the most widely used is the multi UAV mode. Multiple UAVs need to cooperate effectively in the mission to complete the established mission. Among them, due to the “unmanned” characteristics of heterogeneous UAVs, if there is no reasonable task planning in a given task, it will not be able to give full play to the advantages of centralized tasks of multiple UAVs. At the same time, the mutual interference of multiple UAVs in the same space-time dimension may lead to the failure of the original mission [7]. Based on the above situation, we need to focus on the task planning of heterogeneous multi UAV. Task planning of heterogeneous multi UAVs involves two aspects: task allocation and path planning [8]. At present, the task allocation problem of multiple UAVs mainly focuses on task allocation modeling and algorithm [9]. For the former, it is mainly in the multi UAV system, according to the constraints of the given task, on the basis of meeting the task requirements and conditions, to further optimize some objectives, such as shortening the task time and reducing fuel consumption. Based on the above, from the perspective of problem modeling, the classical programming models involved include job shop scheduling problem [10–12]. From the perspective of problem research types, it includes multiple UAVs cooperating to complete a task, jointly attacking a target, multiple UAVs cooperating to complete multiple tasks, that is, heterogeneous UAVs attacking multiple targets, and so on [13]. For example, others have studied the dynamic allocation of distributed autonomous UAVs in cooperative decision-making and strong coupling control; the model involves the strict restriction of time and the constraint of task priority [14]. Some researchers established a multibase vehicle routing mathematical planning model with multiconstraints for the problem of multitask collaborative allocation [15]. For solving the model, first, the exact algorithm such as branch and bound method [16] is proposed. However, with the improvement of model complexity and the need of efficient and fast solution, more effective heuristic algorithms for solving such problems have been proposed, such as genetic algorithm [2], particle swarm optimization [17], and ant colony algorithm [18, 19]. The ant colony optimization algorithm is a new type of simulated evolutionary algorithm. It was initially applied in the field of travel business and can solve major problems of enterprises. Then, it is used to solve assignment problem, scheduling problem, picture coloring problem, routing problem, and so on. The above applications can prove that the ant colony algorithm has strong iterative performance, convergence performance, and wide practical performance. Different evolutionary algorithms are gradually being proposed to solve some problems in the field of UAV technology. For example, other multitarget simultaneous interpreting biological search algorithms [20] are proposed for heterogeneous multi UAVs mission allocation models with different sensor capacities.

In the design of heterogeneous multi UAV, the problems such as path planning need to be further studied. The final result or goal is to generate a specific point-to-point path. Because UAVs perform tasks in space at the same time, the planned path results also require no collision. In multi UAV task planning, different path planning schemes need to be considered in task allocation. Therefore, the path planning problem is considered in the process of building the task allocation model. The task allocation and path planning of multiple UAVs with different combat capabilities and resource constraints are studied, which increases the complexity of task planning research [21]. In order to better realize task allocation and path planning, we need to add random speed to the research model for testing and introduce time window [22]. Before the research, we explored the research of other scholars on UAV continuous mission. In the aspect of solving methods or algorithms of path planning, it mainly includes sampling based method, heuristic method, graph-based search method, and neural network algorithm of computational learning. In the research of path planning for multiple UAVs, researchers proposed an algorithm in the form of decision tree [4]. Elhousari et al. used a new method to solve the model and tested the optimization degree of the algorithm based on multiple data sets [23]. An algorithm that solves the task path planning problem of multiple UAVs was proposed in [24]. Therefore, with the deepening of the research on task planning of heterogeneous multi UAV, evolutionary algorithm and neural network algorithm are proposed to solve the more realistic problem of multi UAV cooperation in a single task or multiple tasks. However, the research on task based on the evolutionary algorithm and neural network is less. Therefore, in order to build and efficiently solve a more practical heterogeneous UAV task allocation and path planning model, this study discusses the task based on ant colony algorithm powered neural network, including model construction, optimization algorithm, and simulation training experiment.

## 2. Heterogeneous Multi UAV Mission Planning Model

### 2.1. Task Planning Problem Description for Heterogeneous Multi UAVs

In terms of time and space dimensions, for the given multitasks in the environment, the problem of selecting and combining different UAV combinations to complete multitasks most efficiently can be regarded as the task planning problem of heterogeneous multi UAV [25].  Figure 1 is taken as an example to show the problem of heterogeneous multi UAV involving six tasks in different base positions, in which “*t*” as the beginning represents the task type. Starting with “*F*” represents the airports with different numbers and types of UAVs, starting with “*n*” represents the no fly zone that may affect the flight of UAVs due to magnetic impact or magnetoelectric interference, and starting with “*L*” represents the possible route of UAVs [26].

Therefore, the task planning problem of heterogeneous multi UAV similar to Figure 1 is to achieve the optimization of the whole heterogeneous multi UAV combat system as far as possible under different task requirements and resource constraints, and its final decision-making goal is to determine the combat task, to optimize the combat system, and to optimize the combat system, the number of combat UAVs, the number of sensors carried by UAVs, the time for each UAV to complete the combat mission, and the flight path for each UAV to perform the combat mission [27].

Based on the above problem description, the parameters defined in this study are as follows: firstly, it is necessary to state the mainly characteristics. The set of multitask location is represented as nodes={0,1,…, *N*}, where is executed only once, and the set of UAVs in different task sizes is represented as No.={1,2,…, *U*}. The set of sensors that can be used in the base is expressed as sensor={1,2,…, *S*}, and the set of no fly zone is expressed as *Q*={*Q*_1_, *Q*_2_,…, *Q*_*q*_}, which is the set of vertices of no fly zone *O*={*O*_1_, *O*_2_,…, *O*_*O*_}. The maximum transportation distance of UAV operation is expressed as *D*_*u*_. It should be noted that for UAV, each UAV can carry multiple sensors. This maximum transportation distance will be affected by the sensors carried by UAV. This reduction is positively proportional to the weight of sensors carried. The maximum load that UAV can bear is *W*_*u*_, the number of sensors that can be used in the base is defined as *E*_*s*_, the weight of sensors is *W*_*s*_, and the reduction factor of the maximum transportation distance *D*_*u*_ with the carrying weight is defined as *C*_*s*_. In addition, the profit of task is defined as *P*_*ts*_, which is mainly related to the profit of completing task *t* and the number of sensors *s* carried by UAV. *P*_*ij*_ represents the path from UAV task *i* to task *j*, *P*_*ij*_ represents the distance from UAV task *i* to task *j*, *β* is a constant, which represents the unit distance cost, and *T*_*tsu*_ represents the time of UAV carrying sensors to complete the task.

Then, due to the complexity of the actual UAV mission situation or environment, this will affect the complexity of the model:

(1) The UAV needs to go to the mission location when performing the mission.
(2) The UAV can maintain the same altitude as far as possible in flight, regardless of the motion path and trajectory of the UAV in three-dimensional space.
(3) The influence of environment on UAV flight can be ignored.
(4) The flight speed of UAV is known constant and does not change.
(5) The flight area of UAV is a regular area, and the no fly area is a regular polygon with multiple vertices. The flight path of UAV can be expressed as a sequence of vertices. The path planning between two vertices that do not pass through the no fly area flies along a straight line, while the path passing through the no fly area is an invalid path. The flight path of UAV is shown in Figure 2 [28].
(6) The kinematics model of UAV follows the classic model proposed by Dubins, which can be expressed as following formulas for this study:
  (1) $$\begin{array}{c} x_{u}=v_{u}\cos\;\phi_{u}, \end{array}$$
  (2) $$\begin{array}{c} y_{u}=v_{u}\sin\;\phi_{u}, \end{array}$$
  (3) $$\begin{array}{c} \phi_{u}=\Omega_{\max}U_{u}. \end{array}$$
In formulas (1)–(3), (*x*_*u*_, *y*_*u*_) represents the position of UAV *u*, *v*_*u*_ is the constant flight speed of UAV mentioned in hypothesis equation (4), *ϕ*_*u*_ is the course of UAV flight, Ω_max_ represents the maximum course change rate of UAV, and *U*_*u*_ represents the condition that UAV steering input satisfies its absolute value less than or equal to 1. In addition, the minimum turning radius *R*_min_ of UAV is expressed as follows:
  (4) $$\begin{array}{c} R_{\min}=\frac{v_{u}}{\Omega_{\max}}. \end{array}$$

### 2.2. Modeling of Heterogeneous Multi UAV Mission Planning Problem

For the heterogeneous multi UAV task planning problem, the objective function is set as two: one is to maximize the overall mission benefits and the other is to minimize the completion time of all tasks. For the goal of maximizing the overall mission benefits, the 0-1 decision variables to be considered in the model are defined as *y*_*tsu*_, *z*_*iju*_, and *f*_*us*_, which, respectively, represent whether the UAV *u* is equipped with sensors *s* to perform task *t*. When the decision variable value is 1, it means yes; otherwise it means no. Whether the UAV *u* moves from the position point of task *i* to the position point of task *j* and whether the UAV *u* is equipped with sensor *s*, 0 and 1 represent the same meaning as before. According to the goal of maximizing the overall system task benefit, the objective function equation is expressed as follows:

(5) $$\begin{array}{c} g_{1}=\max\overset{U}{\underset{u=1}{\sum }}\overset{N}{\underset{t=0}{\sum }}\overset{S}{\underset{s=1}{\sum }}P_{ts}y_{tsu}-\beta \overset{U}{\underset{u=1}{\sum }}\overset{N}{\underset{j:j\neq i}{\sum }}\overset{N}{\underset{i=0}{\sum }}p_{ij}z_{iju}. \end{array}$$

In formula (5), the first half represents the total revenue of UAV carrying sensors to perform tasks in the whole system and the second half represents the total cost of the whole system to complete all tasks. Deducting the cost of completing tasks from the overall revenue is a profit function, while the target function equation (5) is represented to maximize the overall profit.

For the goal of minimizing the total task completion time, the 0-1 decision variable to be considered is *y*_*tsu*_, and the specific definition is the same as the objective function equation (5). Therefore, the objective function of minimizing the total task completion time of the whole system is expressed as the objective function as follows:

(6) $$\begin{array}{c} g_{2}=\min\overset{U}{\underset{u=1}{\sum }}\overset{N}{\underset{t=0}{\sum }}\overset{S}{\underset{s=1}{\sum }}T_{tsu}y_{tsu}. \end{array}$$

The function equation (6) represents the overall task completion time, which needs to minimize the overall task completion time as much as possible.

Next, the constraints of task planning are explained as follows.

For all UAVs *u*,

(7) $$\begin{array}{c} \overset{S}{\underset{s=1}{\sum }}f_{us}\leq M_{u},\;\forall u\in \text{No.}, \end{array}$$

(8) $$\begin{array}{c} \overset{U}{\underset{u=1}{\sum }}f_{us}\leq E_{s},\;\forall s\in \text{sensor.} \end{array}$$

The total weight of each UAV equipped with sensors cannot exceed the limit as follows:

(9) $$\begin{array}{c} \overset{S}{\underset{s=1}{\sum }}f_{us}w_{s}\leq W_{u},\;\forall u\in \text{No}.. \end{array}$$

During the mission, the total flying distance of UAV cannot exceed the maximum flying distance after UAV is equipped with sensors. With the increase in the number of sensors, the maximum flying distance of UAV will be continuously reduced with the coefficient *C*_*s*_, which is expressed as follows:

(10) $$\begin{array}{c} D_{u}-\overset{S}{\underset{s=1}{\sum }}C_{s}f_{us}. \end{array}$$

Based on this, for each UAV *u*, the flight distance constraint is expressed as follows:

(11) $$\begin{array}{c} \overset{N}{\underset{i=0}{\sum }}\overset{N}{\underset{j:j\neq i}{\sum }}p_{ij}z_{iju}\leq D_{u}-\overset{S}{\underset{s=1}{\sum }}C_{s}f_{us},\;\forall u\in \text{No}.. \end{array}$$

Based on this, for each UAV *u*, the flight distance constraint is expressed as follows: in the whole UAV system, each task is executed only once, the effect same as that from task *j* to task *i*, and the required constraint is as follows:

(12) $$\begin{array}{c} \overset{N}{\underset{j=0,i\neq j}{\sum }}z_{iju}\leq 1,\;\forall i\in \text{Nodes},\;\forall u\in \text{No.}, \end{array}$$

(13) $$\begin{array}{c} \overset{N}{\underset{j=0,i\neq j}{\sum }}z_{iju}=\overset{N}{\underset{j=0,j\neq i}{\sum }}z_{jiu},\;\forall u\in \text{No}.. \end{array}$$

For path planning, it is necessary to ensure that the UAV takes off and lands at the base:

(14) $$\begin{array}{c} \overset{N}{\underset{i=0}{\sum }}z_{i0u}=1,\;\forall u\in \text{No.}, \end{array}$$

(15) $$\begin{array}{c} \overset{N}{\underset{i=0}{\sum }}z_{0iu}=1,\;\forall u\in \text{No}.. \end{array}$$

In addition, the constraint that each UAV cannot fly in the no fly zone is expressed as follows:

(16) $$\begin{array}{c} P_{ij}^{u}\cap O=\emptyset ,\;\forall u\in \text{No.}, \end{array}$$

(17) $$\begin{array}{c} P_{io_{1}}^{u}\cap O=\emptyset ,\;\forall u\in \text{No.}, \end{array}$$

(18) $$\begin{array}{c} P_{O_{k}j}^{u}\cap O=\emptyset ,\;\forall u\in \text{No.}, \end{array}$$

(19) $$\begin{array}{c} R_{u}\geq R_{\min}^{u},\;\forall u\in \text{No}.. \end{array}$$

The decision variables of multi UAV mission planning are 0-1 variables; that is, the value can only be 0 or 1:

(20) $$\begin{array}{c} y_{tsu},z_{iju},f_{us}\in \left\{0,1\right\}. \end{array}$$

Based on the above, this paper studies the task allocation, sensor loading, path planning, and other issues when multiple UAVs with different load and kinematics characteristics perform multiple tasks. With the goal of maximizing the revenue of the multi UAV system and minimizing the total task completion time,

(21) $$\begin{array}{c} \left\{\begin{array}{c} \max\overset{U}{\underset{u=1}{\sum }}\overset{N}{\underset{t=0}{\sum }}\overset{S}{\underset{s=1}{\sum }}P_{ts}y_{tsu}-\beta \overset{U}{\underset{u=1}{\sum }}\overset{N}{\underset{j:j\neq i}{\sum }}\overset{N}{\underset{i=0}{\sum }}p_{ij}z_{iju}\\ \min\overset{U}{\underset{u=1}{\sum }}\overset{N}{\underset{t=0}{\sum }}\overset{S}{\underset{s=1}{\sum }}T_{tsu}y_{tsu}\\ \begin{array}{cc} \text{s.t.} & \text{constraint}\left(7\right)-\left(20\right). \end{array} \end{array}\right. \end{array}$$

## 3. Task Planning Solution of Heterogeneous Multi UAV Based on Ant Colony Algorithm Powered Neural Network

### 3.1. Solution of Neural Network Model Based on Ant Colony Algorithm

The main objective of neural network optimization based on the ant colony algorithm is to improve the accuracy of the algorithm proposed for the model and increase the possibility that the solution of the model is close to the global optimal solution rather than the local optimal solution. Aiming at the heterogeneous multi UAV task planning model proposed in this study, the back propagation (BP) neural network algorithm is used in this study. The training of this neural network is mainly based on supervised learning. Through continuous training, the neural network has memory function and memory ability, so it can iterate and optimize the solution more effectively. The design uses the steepest gradient descent method so as to achieve the global optimal solution of task allocation and path planning for multiple UAVs. The specific topological structure of neural network is exhibited in Figure 3.

Specifically, the learning and training of BP neural network are divided into two steps: the forward propagation of signal and the backward propagation of signal. In the first step, the weight values of the input layer and the neurons between the input layer and the hidden layer of the neural network are combined into the hidden layer, such as formula (22), which is used as the input of the hidden layer, and the output of the hidden layer is generated by the activation function after passing through the neural unit in the hidden layer, such as formula (23). Generally, the hidden layer activation function uses a sigmoid function that can convert the real value into a value between 0 and 1, and the formula is expressed as equation (24). Input the weight formula of neurons from the hidden layer, and it is shown in (25). In the output layer, the final output is realized through the linear function as the activation function, such as formula (26).

(22) $$\begin{array}{c} I_{i}=\overset{m}{\underset{h=0}{\sum }}w_{i,h}*x_{h}, \end{array}$$

(23) $$\begin{array}{c} H_{h}=f\left(I_{i}\right), \end{array}$$

(24) $$\begin{array}{c} f\left(y\right)=\frac{1}{1+e^{-y}}, \end{array}$$

(25) $$\begin{array}{c} I_{h}=\overset{N}{\underset{o=0}{\sum }}w_{h,o}*H_{h}, \end{array}$$

(26) $$\begin{array}{c} y_{o}=f\left(I_{h}\right). \end{array}$$

Based on the above formula, we can get the input layer data as the input data of the hidden layer for calculation, and the final output data can be obtained at the output layer after conversion according to the activation function.

In the process of backward propagation, firstly, the deviation between the actual output and the expected value is calculated by absolute value, relative value, or variance, and in this process, the different neurons in the input layer, hidden layer, and output layer are corrected by steepest gradient descent, so as to ensure that the deviation is within a reasonable range or preset range as far as possible. Specifically, the adjustment formulas for the weight value of the steepest gradient descent method are the following formulas:

(27) $$\begin{array}{c} \Delta w_{i,h}=-\eta \frac{\partial \text{error}}{\partial w_{i,h}}, \end{array}$$

(28) $$\begin{array}{c} \Delta w_{h,o}=-\eta \frac{\partial \text{error}}{\partial w_{h,o}}. \end{array}$$

Using the steepest gradient descent method has advantages in solving the complex planning model of heterogeneous UAV task allocation and path planning. The whole architecture of BP neural network includes input layer, hidden layer, and output layer. Sigmoid activation function and linear function are selected for hidden layer and final output function. In addition, in view of the influence of the increase in the number of hidden layer neurons in BP neural network on the training time and the accuracy of the results of the data set, the trade-off between the number of neurons and the length of time and the accuracy of the results are considered, and the general 30 hidden neurons are selected. Specifically, the training process of BP neural network in heterogeneous multi UAV task allocation and path planning is shown in Figure 4.

Although the steepest gradient descent method used in BP neural network is more optimal than the traditional algorithm to achieve the optimal solution, the application of this method will affect the convergence speed of the algorithm and the global optimization of the programming model. Simultaneously, the evolutionary algorithm has the advantages of efficiency and stability in solving the global optimal solution. At the same time, the performance of ant colony algorithm is improved on the basis of previous studies. The BP neural network is further optimized by the ant colony algorithm, and the improvement of the algorithm is realized. To be specific, this method is aimed at optimizing the parameters of neural network.

The optimization and improvement of the genetic algorithm have both the same and different principles with the genetic algorithm. Its essential principle is roughly as follows: for multiple transactions, ants seek the optimal path through mutual communication. Assuming that the number of ants is *m*, in the ant colony algorithm, probability selection is carried out first. The following formula represents the possibility of the ant colony moving from point *i* to point *j*.

(29) $$\begin{array}{c} p_{i,j}=\frac{\tau_{i,j}^{\alpha }\eta_{i,j}^{\beta }}{\sum_{j}\tau_{i,j}^{\alpha }\eta_{i,j}^{\beta }}. \end{array}$$

In formula (29), *τ*_*i*,*j*_^*α*^ represents the pheromone concentration from point *i* to point *j*, *η*_*i*,*j*_^*β*^ represents the expected value of the path from point *i* to point *j*, and *α* and *β* represent the relative importance of pheromone and heuristic factors, respectively. Then, the pheromone is updated. After all the ants cycle from the starting point to all the tasks, many extra nonimportant pheromones will be generated, so the pheromone needs to be updated as follows:

(30) $$\begin{array}{c} \Delta \tau_{i,j}=\underset{m}{\sum }\Delta \tau_{i,j},\\ \Delta \tau_{i,j}\left(t+1\right)=\left(1-\rho \right)\tau_{i,j}\left(t+1\right)+\Delta \tau_{i,j}. \end{array}$$

*ρ* in the formula represents the volatilization coefficient of old pheromone, generally between 0 and 1, and (1 − *ρ*) represents pheromone residue. Then, in order to iterate continuously, the number of training iterations *K* of the first two steps is limited, or the algorithm stops when the error rate reaches a given value. The schematic diagram of the steps is described in Figure 5.

Based on the above, the planning model in this study uses the ant colony algorithm. The final steps are as follows: firstly, the number of nodes in the input layer, hidden layer, and output layer and the number of neurons in the hidden layer of BP neural network are determined, and the expected value is further calculated to prepare for the subsequent deviation calculation. The second is to initialize the parameters including nodes, pheromone concentration, and the number of iterations allowed. Thirdly, the nodes are selected according to the path selection probability of the ant colony algorithm, and the calculated weight parameters are used as the parameters of BP neural network, and then the parameters selected from all ant path sets are also used as the parameters of BP neural network. Then, according to the neural network parameters, using the neural network training data, the result corresponding to the minimum error value is taken as the optimal value of this iteration. When the number of iterations reaches the maximum number, the iteration stops, finds out the optimal value, and updates the pheromone matrix in the ant colony accordingly. The fifth is to calculate whether the minimum error is reached according to the output results. If not, return to the second step for reprocessing. For the specific steps of BP neural network and ant colony algorithm, please refer to Figures 4 and 5.

### 3.2. Experimental Results and Analysis of Neural Network Model Solving Based on Ant Colony Algorithm

By using the training flight data of small high-speed UAV, this paper makes a comparative flight simulation experiment on the neural network heterogeneous multi UAV mission planning technology of the ant colony algorithm. The operating hardware environment of the experimental computer adopts Windows 10 system. The structure of this BP neural network adopts that as shown in Figure 3, and there are 3 hidden layers. The training target is 0.0001, and the learning rate is 0.01. In this paper, the ant colony algorithm is also used, and the population size is 10.80% of the total data and is set as the training set, and the rest is set as the testing data.

In order to verify the effectiveness of task allocation and path planning model of heterogeneous UAV, the test situation is designed, including four heterogeneous UAVs and three sensors in this paper, which have different features. In addition, the number of sensors that UAVs can carry is 2 at most, and there are 4 no flight zones and 30 tasks in the environment, the iteration times in this experiment are set to 5000, and the other parameters are set and modified as per the computed results by this experiment. It is necessary to point out that the maximum of the target (1) is transformed to the minimum for the double objective in this paper, and the weight of each objective function is given 50% to transform the double object into multiobjective for processing. In addition, in order to further verify the stability of the proposed algorithm, 10 repeated experiments have been carried out. The maximum deviation of the 10 programming models for the dual objective function is 1.4%. Therefore, it is considered. The experimental results are shown in Table 1. The path planning of UAV flight is shown in Figure 6.

In this paper, we name the proposed model as ACO-BPNN. In order to verify the performance of the proposed ACO-BPNN model, we compare the proposed method with GA-BPNN and BPNN. The MAE and PERR are used as the metrics to assess the proposed model. The computed results are shown in Figure 7.

As shown in Figure 7(a), the MAE value of ACO-BPNN, GA-BPNN, and BPNN is 4.67, 6.57, and 10.23, respectively. The MAE value of GA-BPNN is increased by 40.7% compared with that of the proposed model, and the MAE value of BPNN is increased by 119.6% compared with that of the proposed model. As shown in Figure 7(b), the PERR value of ACO-BPNN, GA-BPNN, and BPNN is 0.050, 0.086, and 0.120, respectively. The PERR value of GA-BPNN is increased by 72.0% compared with that of the proposed model, and the PERR value of BPNN is increased by 140.0% compared with that of the proposed model. Therefore, from Figure 7, the proposed model ACO-BPNN has a better performance. In order to verify the proposed model more intuitively, we compare the iterations between three different algorithms, as shown in Figures 8–10, respectively. It can be seen from them that the iteration of the proposed model is about 1950 times, and that of GA-BPNN is about 2600 times, and that of BPNN is about 4200 times. Therefore, the iteration speed of the proposed model is better. Overall, in terms of MAE, PERR, and iteration times, the proposed model is better.

The solution process such as ACO-BPNN can avoid falling into local minimum to a great extent. At present, this method has mastered sufficient information on the global level (solution space) and can eliminate most of the local minimum regions. The algorithm proposed in this paper is simulated by the simulation platform developed by MATLAB so as to realize the path display of the algorithm, human-computer interaction control, and so on. Simulation results show that the design scheme is effective and correct and has better dynamic and static performance than the traditional algorithm.

Combined with the fast solving speed of BPNN and the relatively stable solving advantages of ACO, the effect is the best. In addition, compared with other comparative methods, it has further improvement in stability and effectiveness. It is considered that the optimization algorithm can be applied to multi UAV mission planning in practice.

## 4. Conclusion

With the rapid development of UAV technology, how to optimize the UAV flight line and improve the defects in the process of UAV mission is what we need to discuss and study. This paper mainly studies the task planning of heterogeneous multi UAV based on the ant colony optimization neural network algorithm. By analyzing the test cost, the neural network algorithm optimized by ant colony can make effective use of resources and adopt a more effective solution for task planning. In addition to the experimental simulation of heterogeneous multi UAV in the simulation environment, the influence of complex factors on the experimental data is analyzed in the actual environment. Firstly, in addition to the mission planning and design, we also restrict the experimental data according to the load-bearing quantity of UAV, sensor load, no fly area planning, and maximum flight distance. This paper compares the model error and efficiency to some comparative methods and establishes a mathematical model to test it. The experimental results show that the proposed algorithm can improve the operation efficiency of the whole UAV system and shorten the completion time of the total task. It is proved that the algorithm can adapt to the task planning and design of heterogeneous multi UAV and provide support for other aspects of UAV design technology. Subsequently, the heterogeneous multi UAV field is further explored in the complex environment to achieve the best efficiency of the algorithm.

## Figures and Tables

**Figure 1:** Multiple mission planning of heterogeneous multi UAVs.

**Figure 2:** Possible path planning of heterogeneous multi UAVs.

**Figure 3:** The structure of BP neural network.

**Figure 4:** The steps of BP neural network in UAV mission planning.

**Figure 5:** The steps of the ant colony algorithm in parameter optimization of BP neural network.

**Figure 6:** The path planning of multiple mission planning of heterogeneous multi UAVs.

**Figure 7:** Performance comparison of three different algorithms: (a) MAE; (b) PERR.

**Figure 8:** The evolutionary curve of ACO-BPNN.

**Figure 9:** The evolutionary curve of GA-BPNN.

**Figure 10:** The evolutionary curve of BPNN.

**Table 1:** The solution results of multiple mission planning of heterogeneous multi UAVs.

	#1 *S*	#2 *S*	*g*(1)	*g*(2)
*U*_1_	*S*_2_	*S*_3_	1122	2204
*U*_2_	*S*_2_	*S*_1_	1309	2654
*U*_3_	*S*_2_	*S*_3_	944	1849
*U*_4_	*S*_2_	*S*_2_	1224	2406

## Data Availability

The data used to support the findings of this study are available from the corresponding author upon request.
